The article "Session Recommendation Model Based on Context-Aware and Gated Graph Neural Networks" was published in 2021. Journal: Comput Intell Neurosci.

# Session Recommendation Model Based on Context-Aware and Gated Graph Neural Networks

**DOI:** 10.1155/2021/7266960

**Published:** 2021-10-13

**Authors:** Dan Li, Qian Gao

**Affiliations:** School of Computer Science and Technology, Qilu University of Technology (Shandong Academy of Sciences), Jinan 250353, China

## Abstract

The graph neural network (GNN) based approach has been successfully applied to session-based recommendation tasks. However, in the face of complex and changing real-world situations, the existing session recommendation algorithms do not fully consider the context information in user decision-making; furthermore, the importance of context information for the behavior model has been widely recognized. Based on this, this paper presents a session recommendation model based on context-aware and gated graph neural networks (CA-GGNNs). First, this paper presents the session sequence as data of graph structure. Second, the embedding vector representation of each item in the session graph is obtained by using the gated graph neural network (GGNN). In this paper, the GRU in GGNN is expanded to replace the input matrix and the state matrix in the conventional GRU with input context captured in the session (e.g., time, location, and holiday) and interval context (representing the proportion of the total session time of each item in the session). Finally, a soft attention mechanism is used to capture users' interests and preferences, and a recommendation list is given. The CA-GGNN model combines session sequence information with context information at each time. The results on the open Yoochoose and Diginetica datasets show that the model has significantly improved compared with the latest session recommendation methods.

## 1. Introduction

Nowadays, the amount of information on the Internet is exploding. Recommendation system has become an essential tool to ease information overload and improve user experience. Traditional recommendation methods often rely on user profiles and available historical behavior information. However, with the increasing importance of user privacy, it is more and more difficult for the system to get user-related historical information. This requires that the recommendation system make recommendation according to the sequence of users' current interactive sessions. In this case, the recommendation system, which only depends on the sequence of actions in the user's current session to predict the user's next action, is called a session-based recommendation. Sessions are user-site interactions that occur within a given time period [1]. Sessions in a recommendation system usually reflect the user's intentions during this period, such as watching a movie or buying certain goods [2].

The article "Session Recommendation Model Based on Context-Aware and Gated Graph Neural Networks" was published in 2021. Journal: Comput Intell Neurosci.

With the ever-enriching information on the Internet and the ever-increasing ability to collect information, the system has collected more and more available contexts, such as location, time of day, holidays, and preferences. These contextual factors can be used as the basis for modeling user behavior in practice. For example, a user's lunch tends to be more content-rich, while dinner is light. Also, when dining out, preferential meals are more attractive. Therefore, how to apply rich contextual information to session-based recommendations is a challenging and critical issue.

With the rapid development of deep learning technology in recent years, session recommendation algorithms based on deep learning have received more and more attention. Among them, because the graph neural network (GNN) [3, 4] captures the characteristics of dependencies among nodes and gives an excellent performance, GNN has been used to solve session recommendation problems in more and more work in recent years. The current mainstream session recommendation methods focus on the mining of user behavior, which has some drawbacks. One of the main drawbacks is that they do not fully consider and analyze the relevance and contextual information between session items, such as input context related to user decisions, and time interval between user clicks on items.

GNN-based session recommendation can use items as nodes to predict user behavior trends by effectively utilizing project-to-project relationships and content information. Context-aware recommendation methods can integrate multisource and heterogeneous context data to obtain finer-grained item feature information and related relationships. Therefore, the combination of context awareness and session recommendation system has important research value and practical significance.

In this work, we propose a session recommendation model based on context-aware and gated graph neural network, abbreviated as CA-GGNN, which is used to model session information and two kinds of context information in one framework. Compared with GNN, gate graph neural networks (GGNN) introduces gate recurrent unit (GRU) [5] and constructs a message passing model in spatial domain. The output of each layer of the conventional GRU contains the current input information and the previous state information, which are captured by the input matrix and the state matrix, respectively. First, the work of CA-GNN is to model different types of input context information and interval context information to form a specific context matrix associated with the input information dynamically: input matrix and interval matrix. The input matrix represents the scenario information of the external environment when the user makes the current decision, such as the time and place of the day. The interval matrix represents the proportion of the time interval between the current decision and the next decision in the entire session's browsing time. Second, CA-GGNN replaces the constant input matrix and state matrix with input matrix and interval matrix, respectively, and uses a specific context matrix to model the transformation effect of input elements. Finally, this paper uses the time backpropagation algorithm (BPTT) [6] to train the proposed CA-GGNN model. In summary, the main innovations of this work are as follows:

1. This paper proposes a session recommendation model based on context and gated graph neural network. The method includes two types of contexts: input context and interval context. These two contexts, respectively, represent the situation of the external environment when the user participates in the session and the proportion of the time spent by the user browsing each item in the entire session's browsing time.
2. By extending the GGNN loop unit, the state transition of GGNN determined by the defined input, transition, and correlation context is calculated to dynamically model the user interest in the session.

The article "Session Recommendation Model Based on Context-Aware and Gated Graph Neural Networks" was published in 2021. Journal: Comput Intell Neurosci.

The above two innovations of the proposed method are verified by the experiments which are conducted on two real‐world datasets of Yoochoose and Diginetica datasets.

The rest of this paper is organized as follows. The second section discusses the related work. The third section introduces the method and model proposed in this paper in detail. The fourth section gives the experimental results and analysis of the CA-GGNN model. Finally, in the fifth part, the full text is summarized.

## 2. Related Work

In the field of recommendation system, session recommendation has always been a research hotspot. With the introduction of deep learning, Recurrent Neural Network (RNN) has attracted people's attention because of its ability to process sequence data, so it is gradually applied to session recommendation. Hidasi et al. [7] successfully applied GRU to the session recommendation system for the first time. Tan et al. [8] improved Hidasi et al.'s work through optimization methods such as data enhancement technology and setting time threshold. After that, Liu et al. [9] fused the attention network with RNN to avoid the interest offset caused by accidental clicks while capturing the major interests of users in user sessions effectively. Although RNN can handle the dependency between session data, it ignores the dependency of relationship transformation between items in the session.

The article "Session Recommendation Model Based on Context-Aware and Gated Graph Neural Networks" was published in 2021. Journal: Comput Intell Neurosci.

Based on the above problems, Wu et al. [10] used GNN to capture the complex transformation of items and used a soft attention mechanism to integrate user preferences. After that, Xu et al. [11] used the combination of GNN and self-attention network to capture the relationship between adjacent items and the global dependency between items in the session. Yu et al. [12] used users' different interests in different target items to learn the expression of interest vectors that change with the target items. Xu et al. [13] used the complementarity between self-attention network and GNN to enhance recommendation performance. Experiments show that GNN can automatically extract the characteristics of session graph considering rich node connections, which are very suitable for session recommendation.

However, the existing GNN-based recommendation methods still have some limitations. Because they only focus on the session sequence itself, they cannot capture the association relationship between items in the session sequence and the information expressed by the relevant context in the session. GGNN can process the session graph by gating mechanism according to the nature of the session graph and make full use of the dependencies of items in the session. In addition, context awareness has shown good results in the field of recommendation, and its research in the field of GNN-based recommendation needs to be carried out urgently.

Session recording is different from the general behavior sequence. Besides including the user's sequence behavior, it also has two important contextual features: the first feature is the time interval between user behaviors, and the time interval between behaviors has a very important impact on the relationship between user behaviors [14]; the second feature is that the user behavior sequence often contains a large amount of input context information related to user decision-making. These input contexts can better express the user's main intention, which affects the quality of recommendation results.

For the time interval between behaviors, Song et al. [15] added time-gates T1 and T2 to the standard LSTM [16] to separately process the time interval information of the user's click sequence. Liu et al. [17] considered the advantages of modeling context and sequence information at the same time and realized the model of explicit temporal context. In terms of user decision environment, Yuan et al. [18] considered the impact of a variety of context information on recommendation and dynamically modeled user interest by redefining the GRU. Song et al. [19] believe that users' interests are different in each period and are easily affected by friends' interests. Therefore, dynamic graph attention network is used to model the social impact of users' dynamic interests and related contexts. Wang et al. [20] proposed a global context enhanced graph neural network by using the item transformation in the session graph and the global graph, which can better infer the user preferences of the current session.

The article "Session Recommendation Model Based on Context-Aware and Gated Graph Neural Networks" was published in 2021. Journal: Comput Intell Neurosci.

These methods are sufficient to demonstrate that considering both the sequence and context information of the session can improve the recommended performance of the model, and they are also used for reference in this paper. But we still have some extra thoughts about these approaches. On the one hand, for the two context characteristics of session sequence, most context-aware session recommendation methods only use part of the context information in the session as the basis for context recommendation. Therefore, this study considers combining input context and interval context during the session recommendation process to enrich the characteristics of the session.

On the other hand, loop units can handle multidimensional context information and effectively mine the association between session sequences and related contexts. What is unique about GGNN is that it uses GRU loop units to recursively update the embedded vectors of each node in the session graph. Therefore, combining GGNN with context awareness not only enhances the dependencies between items in a session but also fuses context information in a more appropriate way. Based on this, the main work of this paper is to incorporate relevant context information and improve the quality of the GGNN-based session recommendation model.

## 3. Model and Methods of CA-GGNN

This section describes the session recommendation model based on the gated graph neural network and context awareness (CA-GGNN) presented in this paper. This section first gives a statement of the problem and then describes the model definition and optimization of CA-GGNN in this paper.

### 3.1. Problem Definition

In this work, the goal of CA-GGNN is to use GGNN to integrate session sequences and related context information to improve the accuracy of recommendations. A session sequence *s*=[(*v*_1_, *CI*_*v*_1__^*t*_1_^, *CB*_*v*_1__^*t*_1_^),  (*v*_2_, *CI*_*v*_2__^*t*_2_^, *CB*_*v*_2__^*t*_2_^),…, (*v*_*n*_, *CI*_*v*_*n*__^*t*_*n*_^, *CB*_*v*_*n*__^*t*_*n*_^)](*v*_*i*_ ∈ *V*, 1 ≤ *i* ≤ *n*) is arranged from small to large timestamps, where *V*={*v*_1_, *v*_2_,…, *v*_*m*_} for all items involved in all sessions; *CI*_*v*_*i*__^(*t*)^ is the input context representing scenario information such as time and location in the user's current decision; *CB*_*v*_*i*__^(*t*)^ is the interval context, which represents the percentage of the time interval between the timestamp *t*_*k*_ of the current decision and the timestamp *t*_*k*+1_ of the next decision over the entire session's browsing time. The recommended task is to get $\hat{y}=\left\{{\hat{y}}_{1},{\hat{y}}_{2},\ldots ,{\hat{y}}_{m-1},{\hat{y}}_{m}\right\}$ from *s* as input. $\hat{y}$ can be seen as a sorted list. ${\hat{y}}_{j}\left(1\leq j\leq m\right)$ corresponds to the recommended score of an item *j* in this session. The top K items in the list will be the recommended candidates.

The article "Session Recommendation Model Based on Context-Aware and Gated Graph Neural Networks" was published in 2021. Journal: Comput Intell Neurosci.

### 3.2. The CA-GGNN Model

For session recommendation, firstly, this paper obtains two aspects of information based on session sequence. On the one hand, this research uses the information represented by the conversation sequence as a graph structure. On the other hand, this research extracts the input context and interval context, respectively, by using the external environmental factors related to the session and the time interval information between session items. Secondly, each session graph is processed in turn, and the above three kinds of information are input into the extended GGNN to obtain the embedded vector representation based on item nodes in the session graph. Then, the embedded vectors in each session are expressed as global preferences and current interests. Finally, for each session, the model predicts the probability that each item will become the next click item. The overall framework of CA-GGNN is shown in Figure 1.

Figure 1(a) shows the preprocessing of the data in this paper. The data in the dataset are divided into three parts: the input context *ci* consisting of the external environment, the interval context *cb* consisting of the proportion of the time interval between adjacent items in the total session length, and the session graphs by the session sequence. Figure 1(b) shows the extension of this paper to a standard GGNN unit, where *X*(*t*) is the click item at time *t* in the session sequence and *CI*(*t*) and *CB*(*t*) are adaptive input matrices and interval matrices generated by the input context and interval context corresponding to *X*(*t*). When the GGNN loop is over, the embedded vector *v*_*i*_ of each item node can be obtained. Figure 1(c) shows the recommended process. This paper uses the soft attention mechanism to integrate user preferences to gain long-term interest and uses the last item in the session sequence as the user's short-term interest. A vector representation of the session sequence is got through a linear connection and used as the basis for recommendation.

### 3.3. Gated Graph Neural Network

GGNN considers both the structure information of the graph and the state information of each node at each time to generate an accurate representation of the node vector. GGNN can construct a more reliable session representation than RNN. Specifically, the learning update function for the graph **G** node vector *v*_*i*_ [9] is shown in the following formulas:

(1) $$\begin{array}{c} a_{v_{i}}^{\left(t\right)}=A_{V:}{\left[h_{v_{1}}^{\left(t-1\right)},\ldots ,h_{v_{n}}^{\left(t-1\right)}\right]}^{T}H+b, \end{array}$$

(2) $$\begin{array}{c} r_{v_{i}}^{\left(t\right)}=\sigma \left(a_{v_{i}}^{\left(t\right)}W_{r}+h_{v_{i}}^{\left(t-1\right)}U_{r}\right), \end{array}$$

(3) $$\begin{array}{c} z_{v_{i}}^{\left(t\right)}=\sigma \left(a_{v_{i}}^{\left(t\right)}W_{z}+h_{v_{i}}^{\left(t-1\right)}U_{z}\right), \end{array}$$

(4) $$\begin{array}{c} {\tilde{h}}_{v_{i}}^{\left(t\right)}=\tanh\left(a_{v_{i}}^{\left(t\right)}W+\left(r_{v_{i}}^{\left(t\right)}⊙h_{v_{i}}^{\left(t-1\right)}\right)U\right), \end{array}$$

(5) $$\begin{array}{c} h_{v_{i}}^{\left(t\right)}=\left(1-z_{v_{i}}^{\left(t\right)}\right)⊙h_{v_{i}}^{\left(t-1\right)}+z_{v_{i}}^{\left(t\right)}⊙{\tilde{h}}_{v_{i}}^{\left(t\right)}, \end{array}$$

where *h*_*v*_*i*__^*t*^ represents the implicit vector of the node and *a* is the adjacency matrix based on the session graph. Formula (1) shows the steps of transmitting information between different nodes in the diagram. Formulas (2) to (5) are information transmission methods similar to GRU, which predicts the output results of a given node at each time step *T* and then updates the hidden state of each node. The implicit vector representation of each item in the session can be got by repeating the update until convergence, where *z*_*v*_*i*__^*t*^ and *r*_*v*_*i*__^*t*^ represent update gate and reset gate and *σ*(·) is usually selected as S-type function [10] as shown in

(6) $$\begin{array}{c} \sigma \left(x\right)=\exp\left(\frac{1}{1+e^{-x}}\right). \end{array}$$

Although GGNN has achieved satisfactory results in session modeling, it still has some limitations because it ignores the assistive role of various contextual information in session recommendation. To address these issues, this paper attempts to incorporate contextual information into GGNN-based session modeling.

The article "Session Recommendation Model Based on Context-Aware and Gated Graph Neural Networks" was published in 2021. Journal: Comput Intell Neurosci.

### 3.4. Extension of GGNN Units

From the above analysis, we can see that formulas (3)–(5) cannot meet the need for fusing contextual information. Therefore, this paper extends the existing GGNN cycle elements. The input context and interval context presented in this paper are incorporated into the regular GRU cell. This makes the process of session recommendation dependent not only on session sequence information but also on the session sequence and related context information. The specific extension methods are as follows.

As you can see from Section 3.2, formula (4) represents the hidden state of the items in the session sequence at each time and consists of the current node item representing *a*_*v*_*i*__^(*t*)^ and the hidden state of the previous node *h*_*v*_*i*__^(*t* − 1)^. *W* and *U* are derived from learning historical data and are used to simulate the recursive signal representation of an item in a continuous hidden state. Therefore, this paper simplifies the representation of the hidden state of the item at time *t* to

(7) $$\begin{array}{c} {\tilde{h}}_{v_{i}}^{\left(t\right)}=\tanh\left(a_{v_{i}}^{\left(t\right)}W+h_{v_{i}}^{\left(t-1\right)}U\right). \end{array}$$

In this case, we consider incorporating the adaptive input matrix and transition matrix presented in this paper into the *W* and *U* of formula (6). This not only enables GNN to enhance the correlation between adjacent items but also adds context to the sequence prediction during the update iteration. Using GGNN to fuse input and interval contexts eliminates or reduces the negative impact of ignoring the relevance of adjacent items. Thus, the hidden state of the output of each item node in GGNN at time *t* can be expressed as

(8) $$\begin{array}{c} {\tilde{h}}_{v_{i}}^{\left(t\right)}=\tanh\left(a_{v_{i}}^{\left(t\right)}W_{CI_{v_{i}}^{\left(t\right)}}+h_{v_{i}}^{\left(t-1\right)}U_{CT_{v_{i}}^{\left(t\right)}}\right), \end{array}$$

where *a*_*v*_*i*__ is the embedded vector associated with the item *i*; *W*_*CI*_ is the input context weight matrix for time *t*, which represents the environmental context associated with the current input item, such as time, place, holiday, and preferences; and *U*_*CT*_ is a specific interval context weight matrix that represents the time interval between two adjacent items in a session. However, we cannot learn a specific interval context matrix for each possible continuous interval value. Therefore, this paper replaces the information about the time interval between two items with the proportion of the total session duration of the item's browsing time.

We consider that when users browse items, they spend more time on items that are more interesting than items that are not interesting or that have missed points. Therefore, this research replaces the time interval information between two items with the percentage of each item's browsing time over the entire session. This can indicate the relevance of the user's current click-through item to the user's current interest. For example, users browse items *v*_1_, *v*_2_, and *v*_3_ for 45 s, 360 s, and 60 s in session s1 and for 240 s, 300 s, and 360 s in session *s*_2_. Obviously, the users' interest in item *v*_3_ is much greater in session *s*_1_ than in session *s*_2_. Therefore, this paper uses the standard score [21] *z*_*v*_*i*__ to represent the relative position of the item browsing time information in the session and uses the S-type function [10] to normalize the standard score, as shown in

(9) $$\begin{array}{c} z_{v_{i}}=\frac{t_{v_{i}}-{\bar{t}}_{s,v}}{T}, \end{array}$$

(10) $$\begin{array}{c} b_{v_{i}}=\frac{1}{1+e^{-z_{v_{i}}}}. \end{array}$$

Thus, formula (7) can be rewritten as

(11) $$\begin{array}{c} {\tilde{h}}_{v_{i}}^{\left(t\right)}=\tanh\left(a_{v_{i}}^{\left(t\right)}W_{CI_{v_{i}}^{\left(t\right)}}+h_{v_{i}}^{\left(t-1\right)}U_{CB_{v_{i}}^{\left(t\right)}}\right), \end{array}$$

where *U*_*CB*_ represents a specific interval context matrix, which is used to represent the proportion of item *v*_*i*_ in its session.

The article "Session Recommendation Model Based on Context-Aware and Gated Graph Neural Networks" was published in 2021. Journal: Comput Intell Neurosci.

In addition, formula (3) represents the update gate *z*_*v*_*i*__^(*t*)^ in the cycle unit, which is mainly used to determine the proportion of historical information and current information to be transmitted. This paper holds that the update gate not only can depend on the current input and the information of the previous hidden state but also must consider the current context. Therefore, this paper rewrites the update door as

(12) $$\begin{array}{c} z_{v_{i}}^{\left(t\right)}=\sigma \left(a_{v_{i}}^{\left(t\right)}W_{z}+h_{v_{i}}^{\left(t-1\right)}U_{z}+C_{I,B}^{\left(t\right)}V_{Z}\right), \end{array}$$

where *C*_*I*,*B*_^(*t*)^ represents the relevant context of the item at time *t* and *V*_*Z*_ is the corresponding weight matrix.

### 3.5. Session Vector Representation

This paper uses the representation method of session vector *S* proposed by Wu et al. [10]. First, take the last clicked item in the session as the user's current preference *s*_*s*_ and the previous clicked item as the long-term preference *s*_*l*_. Then, the soft attention mechanism is used to measure the priority of each item compared with the current preference. It is expressed as

(13) $$\begin{array}{c} \alpha_{i}=q^{T}\sigma \left(W_{1}V_{n}+W_{2}V_{i}+c\right), \end{array}$$

(14) $$\begin{array}{c} s_{l}=\sum_{i=1}^{n}\alpha_{i}V_{i}, \end{array}$$

(15) $$\begin{array}{c} S=W_{3}\left[s_{s};s_{l}\right], \end{array}$$

where *α*_*i*_ is the attention factor that measures item priority, *V*_*i*_ is the embedded vector for each item in the session, and the parameters *q* ∈ *ℝ*^*d*^, and *W*_1_ and *W*_2_ are used to adjust the weight of the embedded vector for the item.

### 3.6. Recommendation Layer

After the model training, we can get the current item's embedded vector *V*_*i*_ and the session's embedded vector *S*. For each candidate's final recommended probability, the point product is used first, and then the S-type function is [10] used to obtain the output vector $\hat{y}$. $\hat{y}$ is expressed as

(16) $$\begin{array}{c} {\hat{y}}_{i}=\text{soft}\max\left(S^{T}V_{i}\right), \end{array}$$

where ${\hat{y}}_{i}\in \hat{y}$ indicates the probability that item *V*_*i*_ will be the next click on an item in the current session.

The article "Session Recommendation Model Based on Context-Aware and Gated Graph Neural Networks" was published in 2021. Journal: Comput Intell Neurosci.

Then, the cross-entropy loss function [22] is used to measure the final prediction result, as shown in

(17) $$\begin{array}{c} ℒ\left(\hat{y}\right)=-\sum_{i=1}^{m}y_{i}\log\left({\hat{y}}_{i}\right)+\left(1-y_{i}\right)\log\left(1-{\hat{y}}_{i}\right), \end{array}$$

where *y* is a one-hot coded vector representing the basic true value of the item.

Finally, the CA-GGNN model is trained using the time reverse propagation algorithm BPTT [6].

## 4. Experimental Results and Analysis

In this section, we study the effectiveness of CA-GGNN in session recommendation through experiments. First, we describe the experimental settings for this paper. Then, the proposed CA-GGNN model is compared with other methods, and a comparison experiment is carried out for input context and interval context. Finally, the different experimental settings are analyzed in detail.

### 4.1. Datasets

This experiment was conducted on two real-world datasets with rich contextual information. The Yoochoose dataset is a public dataset from RecSys Challenge 2015 that contains records of user behavior over a six-month period. There are 9249729 items and 33003994 user click records. The Diginetica dataset, from CIKM Cup 2016, contains 43097 items totaling 204771 user click records.

In order to ensure the fairness of the experiment, this paper filters out all items with a session length of 1 and occurrences less than 5 times in both datasets, referring to the practices of Li et al. [23] and Liu et al. [9]. This is because data that has a short session length or fewer item browses is not valuable to use. In addition, the dataset is also split. For Yoochoose datasets, this paper uses the last day's data as the test set and other data as the training set. For the Diginetica dataset, the last seven days are used as the test set and the rest as the training set. The Yoochoose dataset is too large to be trained and tested by the model. Therefore, the dataset is divided into 1/64 and 1/4 datasets using the commonly used segmentation method. Statistics about the dataset are shown in Table 1.

Based on the context information in both datasets, this paper extracts the environment context and the interval context to implement the CA-GGNN model presented in this paper. First, this paper extracts different kinds of contexts on two datasets using timestamp information. On the Yoochoose dataset, this paper extracts three types of input context information, a total of 210 input context values, including seven days a week, six time periods in a day, and the type of user's click context (such as preference, type of click item). On the Diginetica dataset, two input contexts are extracted: seven days a week and six periods in a month. Therefore, there are 42 input context values in the Diginetica dataset. Secondly, this paper takes the interval context as the ratio of the browsing time of each item in the sequence to the total session length. In order to facilitate the modeling of interval context, we normalize the interval context. We divide the interval context in the two datasets into 10 types, which can effectively prevent the problem of data sparsity. Therefore, there are 10 interval context values for both datasets.

The article "Session Recommendation Model Based on Context-Aware and Gated Graph Neural Networks" was published in 2021. Journal: Comput Intell Neurosci.

### 4.2. Evaluation Indices

P@K [24] (precision) is used to measure the accuracy of the prediction structure in the session recommendation system, indicating the proportion of the top K items in the list of recommendation results to the correct sample.

MRR@K [25] (mean reciprocal rank) means the average reciprocal rank. This method builds on the P@K method and adds the impact of item location. The higher the item's position in the list of recommended results, the smaller the value and vice versa. The value is 0 when the item is not among the first K recommended items.

In this paper, *K* = 20 is used for evaluating the model, because in the actual scenarios of most session recommendation systems, most users only focus on the recommendations that appear on the first page.

## 5. Parameter Settings

The parameters of the model are set as follows: the dimension of the embedded vector and the number of GRU are set to 100, learning rate = 0.001, learning rate decay rate = 0.1, batch size = 100, and the number of iterations = 30. All weight matrices initialize all parameters with a Gaussian distribution with a mean of 0 and a standard deviation of 0.1. The model uses the cross-entropy loss function and the Adam optimization method to solve the model parameters.

### 5.1. Comparison Algorithms

To evaluate the validity of the proposed model, we studied the validity of CA-GGNN from different perspectives and compared the model with the following eight representative models.

  POP and S-POP [7]: they are popularity-based prediction methods used to recommend the most frequently occurring commodities in a dataset.
  BPR-MF [26]: it is one of the most commonly used matrix algorithms at present used to optimize the pairwise sorting loss function mainly through the random gradient descent method.
  Item-KNN [27]: based on the KNN algorithm of an item, the similarity of an item is mainly calculated according to its cooccurrence in session recommendation, and it is recommended through recall and most similar items in session.
  FPMC [28]: it is a sequence prediction method based on Markov chain and matrix factorization. This method is mainly used in the recommendation system to predict the likelihood that unknown items will be of interest to users and then to drain the recommendation list of items.
  GRU4REC [7]: this is the first time that RNN is applied to the session recommendation task. RNN is used to model the click sequence of users, and samples are taken according to the popularity of items. The sampling results are divided into positive and negative samples, and the rank-based loss function is used.
  NARM [23]: based on the RNN based session recommendation model, the attention mechanism is used to capture the user's purpose in the current session from the hidden state.
  STAMP [9]: it introduces both memory and attention mechanisms, considering user's long-term/short-term interests. It is used to reduce the impact of interest drift on the recommended results by increasing the weight of short-term interests.
  SR-GNN [10]: it sets session sequence behavior as graph data, captures transfer patterns between items through GNN, and captures user interest using attention mechanism.
  TAGNN [12]: it represents a target attention graph neural network based on session recommendation. Target-aware attention can adaptively activate users' different interests in different target objects and learn about the dynamic changes of users' intentions.
  DGTN [29]: it presents a two-channel graph conversion network using the conversion relationship between objects. This method integrates the target session and neighbor session into one graph and uses channel-aware propagation to explicitly encode the session signal of the item into the embedding vector of the item.

The article "Session Recommendation Model Based on Context-Aware and Gated Graph Neural Networks" was published in 2021. Journal: Comput Intell Neurosci.

### 5.2. Overall Comparison

To verify the effect of the CA‐GGNN model on the Yoochoose1/64, Yoochoose1/4 and Diginetica datasets, this article shows the comparative experiment results of CA‐GGNN and other models.

From Table 2, it can be seen that the traditional session recommendation methods, BPR-MF, Item-KNN, and FPMC, have significantly improved the benchmark performance of POP. This indicates that the sequence information of the session sequence has more influence in the scenarios recommended by the session. Nonetheless, S-POP performs better than BPR-MF and is more stable, which demonstrates the importance of context information for session recommendation. Among all the comparison methods, the method based on deep learning has the best performance, which reflects the superiority of deep learning technology in capturing user's interests. However, for all indicators, the results of the CA-GGNN model presented in this paper perform best on the three datasets. The improvement range of P@20 is about 1.31%–71.6%, and the relative improvement range of MRR is about 1.42%–32.61%. These improvements demonstrate the need to model both input and interval contexts. Through deep learning technology, we can better grasp the complex and hidden connections of user's interests, whereas the contextual information in the session not only helps the model to cope with noisy session data effectively but also enhances the stability and robustness of the model, which can further improve the accuracy of recommendations.

#### 5.2.1. Context Impact

To verify the usefulness of context, this paper compares the CA-GGNN model with the SR-GNN model [12] without context information. On three datasets, Yoochoose1/64, Yoochoose1/4, and Diginetica, the P@20 and MRR@20 of the CA-GNN and SR-GNN models are compared as shown in Figure 2.

From Figure 2, we can see that, in the three datasets, the accuracy of the CA-GGNN model and SR-GNN model does not fluctuate significantly after the fifth epoch, and the model tends to be stable. Since then, the CA-GGNN model has certain improvement compared with the SR-GNN model, the gap is obvious and stable, and the specific results are shown in Table 2. This indicates that the integration of relevant contextual information in session recommendation really improves the effectiveness of the model. From the trend of P@20 and MRR@20 in Figure 2, the SR-GNN model shows significant fluctuations during the first four iterations, while the CA-GGNN model shows a steady upward trend. It can be seen that the CA-GNN model is more robust and less susceptible to other factors when considering both session sequence information and context information. Overall, the model in this paper does improve the effectiveness of the model by incorporating contextual information about user decisions. The improvement is more significant on the datasets with large data volumes of Yoochoose1/4 and Diginetica.

#### 5.2.2. Impact Analysis in Two Contexts

The impact of context information on session recommendation is also divided into three aspects: (1) only input context CA-GGNN model (only input); (2) CA-GGNN model with only interval context (only interval); (3) CA-GGNN model with both input and interval contexts (input and interval).  Figure 3 shows the results with these three different contextual strategies.

The article "Session Recommendation Model Based on Context-Aware and Gated Graph Neural Networks" was published in 2021. Journal: Comput Intell Neurosci.

The results in Figure 3 show that the CA-GGNN model achieves the best performance among the three contextual scenarios. The CA-GGNN model improves P@20 by about 0.61%, 2.3%, and 0.1%, and MRR@20 by about 1.2%, 0.81%, and 0.38% compared with the model with only input context. Compared with the model that only integrates interval context, the CA-GGNN model improves P by about 1.54%, 1.31%, and 0.25%, and MRR improves by about 0.91%, 0.21%, and 0.44%. This indicates that both kinds of contextual information are important for session recommendation and have different roles in different situations of recommendation.

### 5.3. Comparison with Other Latest GNN-Based Session Recommendation Models

With the development of model research, GNN-based session recommendation has received more and more attention. Therefore, we consider whether the CA-GGNN model has better recommended performance than other latest GNN-based session recommendation models. We compare the proposed CA-GGNN model with the latest GNN-based session recommendation model “TAGNN” and “DGTN.” The experimental results are shown in Table 3.

From Table 3, we can see that the experimental results of CA-GGNN are higher than those of TAGNN and DGTN. Both TAGNN and DGTN models consider the complexity of capturing project relationships in a session using GNN and model transformational relationships between users or projects. However, they both ignore the important impact of contextual information in the session on the recommendation process. Through analysis, we can see that context information is one of the important factors that affect session recommendation. In addition, the CA-GNN model improves significantly on Yoochoose1/4 and Diginetica datasets. This indicates that the CA-GGNN model can obtain more accurate recommendation results in numerous recommended scenarios.

In summary, the CA-GGNN model proposed in this paper can effectively model the context information in the session. After fusing the relevant context information, the CA-GGNN model is more stable and the accuracy is further improved. Moreover, when the amount of data is large, the effect of model improvement is more obvious. This shows that it is necessary to introduce context information into the process of session recommendation.

## 6. Conclusion

Currently, most of the recommended methods for sessions only use sequence information in the session, without considering the impact of relevant context information on session recommendation. To solve this problem, this paper presents a novel method, which is a session recommendation model based on context-aware and gated graph neural network. In this paper, the session sequence is represented by a graph structure, fully considering the internal relationship between session items. Then, the input context and interval context associated with the session sequence are incorporated into the recommendation process by extending the GGNN unit. This enables the model to cope with complex real-world situations with stronger robustness. The comprehensive experimental results show that the method proposed in this paper is superior to other advanced methods.

The article "Session Recommendation Model Based on Context-Aware and Gated Graph Neural Networks" was published in 2021. Journal: Comput Intell Neurosci.

## Figures and Tables

**Figure 1:** Overall framework of CA-GGNN. (a) Data preprocessing. (b) Extension of GGNN. (c) Recommendation process.

**Figure 2:** Comparison of CA-GGNN and SR-GNN experimental results.

**Figure 3:** Impact of different contexts on recommendations.

**Table 1:** Dataset statistics.

	Yoochoose1/4	Yoochoose1/64	Diginetica
Train	5917745	369859	719470
Test	55898	55898	60853
Items	29618	16766	43097

**Table 2:** Performance comparison of different models on two datasets (%).

Method	Yoochoose1/64		Yoochoose1/4		Diginetica	
	P@20	MRR@20	P@20	MRR@20	P@20	MRR@20
POP	6.71	1.65	1.33	0.30	0.89	0.23
S-POP	30.44	18.35	27.08	17.75	21.06	13.68
BPR-MF	31.31	12.08	3.40	1.57	5.24	1.98
Item-KNN	51.60	21.81	52.31	21.70	35.75	11.57
FPMC	45.62	15.01	—	—	26.53	6.95
GRU4REC	60.64	22.89	59.53	22.60	29.45	8.33
NARM	68.32	28.63	69.73	29.23	49.70	16.17
STAMP	68.74	29.67	70.44	30.00	45.64	14.32
SR-GNN	69.53	30.41	70.90	30.43	49.70	16.31
CA-GGNN	**70.84**	**31.83**	**72.93**	**32.91**	**51.12**	**18.48**
Improve	1.31	1.42	2.03	2.48	1.42	2.17

Bold shows the experimental result of the model proposed in this paper. The results of FPMC experiments on Yoochoose1/4 datasets were not published because the FPMC model could not be initialized due to insufficient memory.

**Table 3:** Comparison of the experimental results of CA-GGNN with TAGNN and DGTN (%).

Method	Yoochoose1/64		Yoochoose1/4		Diginetica	
	P@20	MRR@20	P@20	MRR@20	P@20	MRR@20
TAGNN	70.17	30.46	71.05	30.96	50.02	17.18
DGTN	70.21	31.08	71.38	31.37	50.35	17.33
CA-GGNN	**70.84**	**31.83**	**72.93**	**32.91**	**51.12**	**18.48**
Improve	0.63	0.75	1.55	1.18	0.77	1.15

Bold shows the experimental result of the model proposed in this paper.

## Data Availability

The Yoochoose and Diginetica datasets used to support the findings of this study have been deposited in the GitHub repository. Copies of these data can be obtained free of charge from https://github.com/Arrietti-li/Dataset/tree/e2cdcfcce7ed0df3fbcfb8ec6a1692676d23f638.
